# Repeated allergen exposure reduce early phase airway response and leukotriene release despite upregulation of 5-lipoxygenase pathways

**DOI:** 10.1186/2045-7022-2-7

**Published:** 2012-03-22

**Authors:** Zhi-Hua Cui, Madeleine Rådinger, Margareta Sjöstrand, Jan Lötvall

**Affiliations:** 1 Krefting Research Centre, Department of Internal Medicine and Clinical nutrition, Institute of Medicine, University of Gothenburg, Gothenburg, Sweden; 2 Gilead Sciences, Inc., 199 East Blaine Street, Seattle, WA 98102, USA

**Keywords:** Guinea pig, Allergen exposure, Cholinergic responsiveness, Early phase airway response, Plasma exudation, 5-lipoxygenase, Cyclooxygenase

## Abstract

**Background:**

Allergen induced early phase airway response and airway plasma exudation are predominantly mediated by inflammatory mast cell mediators including histamine, cysteinyl leukotrienes (cysLTs) and thromboxane A2 (TXA2). The aim of the present study was to evaluate whether repeated allergen exposure affects early phase airway response to allergen challenge.

**Methods:**

A trimellitic anhydride (TMA) sensitized guinea pig model was used to investigate the effects of low dose repeated allergen exposure on cholinergic airway responsiveness, early phase airway response and plasma exudation, as well as local airway production of mast cell derived cysteinyl leukotrienes and thromboxane B2 (TXB2) after allergen challenge.

**Results:**

Repeated low dose allergen exposure increased cholinergic airway responsiveness. In contrast, early phase airway response and plasma exudation in response to a high-dose allergen challenge were strongly attenuated after repeated low dose allergen exposure. Inhibition of the airway response was unspecific to exposed allergen and independent of histamine receptor blocking. Furthermore, a significant reduction of cysteinyl leukotrienes and TXB2 was found in the airways of animals repeatedly exposed to a low dose allergen. However, in vitro stimulation of airway tissue from animals repeatedly exposed to a low dose allergen with arachidonic acid and calcium ionophore (A23187) induced production of cysteinyl leukotrienes and TXB2, suggesting enhanced activity of 5-lipoxygenase and cyclooxygenase pathways.

**Conclusions:**

The inhibition of the early phase airway response, cysteinyl leukotriene and TXB2 production after repeated allergen exposure may result from unresponsive effector cells.

## Introduction

Early phase airway response to allergen and airway plasma exudation are predominantly mediated by inflammatory mediators including histamine, cysteinyl leukotrienes (cysLTs) and thromboxane A2 (TXA2) [1-3] released from mast cells in the response to allergen challenge [4-7]. In asthmatic patients, the concentrations of cysLTs and TXA2 are increased in plasma, urine and BAL fluid during asthma exacerbation and after experimental allergen challenges [8-11]. Thus, these mediators can induce both airway constriction and airway plasma exudation in several species [3,12-14]. Production of these mediators needs the substrate arachidonic acid and enzymes such as 5-lipoxygenase (5-LO) and cyclooxygenase (COX) [15]. Furthermore, mast cell responsiveness involve expression and binding of allergen to the high affinity IgE-receptor (FcεRI) and subsequent activation of intracellular signaling molecules activating the 5-LO and COX pathway [16-19].

Repeated or chronic exposure to low doses of allergen, such as house-dust mite, animal dander, or some occupational allergen is quite common in real life. Evidence obtained from human subjects and animal models suggest that repeated allergen exposure may induce non-specific bronchial hyperresponsiveness (BHR) and airway inflammation [20-22]. However, the effect of repeated exposure to allergen on the early phase airway response however is not clear. Thus, in the current study, we hypothesize that repeated allergen exposure may reduce early phase airway response, since patients allergic to cat repeatedly exposed to low doses of cat allergen prior to high dose allergen challenge, displayed a attenuated late phase response despite existing bronchial hyperresponsiveness [23]. Therefore, the aim of the present study was to evaluate whether repeated exposure to allergen affects early phase airway response to allergen and further elucidate the possible mechanisms. Thus, in the present study, we utilized a trimellitic anhydride (TMA) sensitized guinea pig model. TMA is an occupational small molecular allergen widely encountered in plastic industry. Furthermore, it is known that skin contact and inhalation of TMA can stimulate the immune system and thus induce asthma in humans [24]. In the present study, we repeatedly exposed sensitized guinea pigs to allergen (TMA), prior to the high dose challenge and evaluated cholinergic bronchial responsiveness and specific early phase airway responses to allergen. We also tested the possible mechanisms behind the changes of early phase airway response, including the levels of cysLTs and TXB2 in airway, activity of 5-LO and COX pathways, as well as the activity of protein tyrosine kinase Lyn, one of intracellular signaling molecules downstream FcεRI.

## Materials and methods

### Allergen sensitization and exposure

Male Dunkin Hartley guinea pigs (initial weight 200-250 g) were obtained from HB Sahlins Försöksdjurfarm, Malmö, Sweden. Guinea pigs were sensitized by intradermal injection of a suspension of 3, 1, and 0.1 mg of TMA in 0.1 ml corn oil on day 1, 10 and 20, respectively (Figure 1). Intradermal injection (i.d.) of corn oil was used as control substance in non-sensitized animals. In double sensitization experiments, animals were sensitized as above but also administered 0.3 mg ovalbumin in 0.1 ml PBS i.d. On day 30 to 34, animals were exposed to an aerosol of TMA conjugated to guinea pig serum albumin (TMA-GPSA). Guinea pigs were exposed either to a high dose (0.15% TMA-GPSA) once for 15 min (day 34), or to low doses (0.03% TMA-GPSA) for 15 min each day on 5 consecutive days (day 30-34), in a Plexiglas chamber (Figure 1). Aerosol of the vehicle (PBS) was used as control. The aerosols were generated by a compressed air jet nebulizer (Maxin MA2, Clinova Medical AB, Malmö, Sweden; mean mass diameter < 3 μm in water). Pyrilamine (10 mg/kg, i.p.) was used 30 min before aerosol exposure to block the effects of histamine to minimize the potential fatal airway responses. This study was approved by the animal ethics committee in Göteborg. Dnr 88/98.

**Figure 1:** **Experimental design**. Briefly, animals were sensitized by intradermal injection of a suspension of 3, 1, and 0.1 mg of TMA in 0.1 ml corn oil on day 1, 10 and 20, respectively. In double sensitization experiments, animals were sensitized as above but also administered 0.3 mg ovalbumin in 0.1 ml PBS by intradermal injection. Animals were exposed to an aerosol of PBS or TMA conjugated to guinea pig serum albumin (TMA-GPSA) on day 30 to 34. One group of animals was exposed to PBS on day 30-33 followed by a high dose TMA-GPSA (0.15%) exposure once for 15 min on day 34. One group of animals was exposed to a low dose TMA-GPSA (0.03%) for 15 min each day on 5 consecutive days. ACh responsiveness was evaluated 24 hours after the last exposure. The early airway response to TMA-GPSA was measured one hour after the completion of the ACh responsiveness (some changes were made on day 35 for other experiments, see study design/protocol section). Bronchial alveolar lavage (BAL) fluid was taken immediately after the assessment of early airway response.

### Study design

Animals were divided into four groups (7-12 in each group). Group 1 was not sensitized (i.d. corn oil), and was sham-exposed to PBS on 5 consecutive days. Group 2, 3, and 4 were sensitized to TMA. Group 2 was exposed to PBS on 5 consecutive days; group 3 was exposed to PBS on 4 consecutive days, followed by a single high dose of TMA-GPSA (0.15%) exposure; group 4 was exposed to low dose of TMA-GPSA (0.03%) on 5 consecutive days. The total dose of allergen received by animals of group 3 and 4 was exactly the same. ACh responsiveness was evaluated 24 hours after the last exposure. The early airway response to TMA-GPSA was measured one hour after the completion of the ACh responsiveness. BAL fluid was taken after the early airway response measurement, for evaluation of inflammatory cells and levels of LTC4/D4/E4, TXB2 and PGE2 (Figure 1).

### Cholinergic airway responsiveness

Anaesthetized and ventilated guinea pigs were provoked with inhaled aerosol of acetylcholine (ACh) (1 × 10^-5^, 3 × 10^-5^, 1 × 10^-4 ^and 3 × 10^-4 ^M; 10 ml/kg for 20 inhalations) at a 10-min interval until RL increased at least 500% above the baseline. Aerosol was generated by an ultrasonic nebulizer (Pulmo-Sonic Model 2511, The DeVilbiss Co., Somerset, PA, U.S.A.) and driven by a ventilator. Lung resistance (RL) was measured as previously described [22] immediately after each ACh provocation for 10 min. A dose-response curve was constructed, and cholinergic airway responsiveness was expressed as provocative concentration of ACh, which increased RL 500% above the baseline (-Log PC_500_). Ten minutes before ACh provocation, animals were pretreated with pyrilamine (5 mg/kg, i.v.), propranolol (1 mg/kg, i.v), and suxamethonium 5 mg i.v.).

### Early phase airway response to allergen

One hour after the completion of ACh assessment, animals were challenged with intratracheal instillation of 250 μg TMA-GPSA in 50 μl PBS. Lung resistance was measured for 10 min. The immediate airway response was expressed as area under the curve (AUC) of RL from 0 to 10 minutes for statistical analysis.

#### Specificity of early phase airway response to exposed allergen

To evaluate the specificity of early phase airway response to exposed allergen, we sensitized animals of three groups (7 in each group) with both TMA and OVA. Group 1 was exposed to PBS, group 2 to 0.03% TMA-GPSA, and group 3 to 0.03% OVA on five consecutive days. Early phase airway response and Evans blue dye exudation to OVA challenge were evaluated 24 hours after the last exposure.

#### Analysis of Evans blue dye exudation

Evans Blue dye (20 mg/kg) was injected i.v. over one minute, two minutes before allergen challenge. Animals were sacrificed by an over-dose of anaesthesia after the assessment of airway obstruction. The thoracic cavity was opened and systemic and pulmonary circulation was perfused with 100 ml PBS, respectively. The trachea, main bronchi, proximal intrapulmonary airways (PIA), distal intrapulmonary airways (DIA) was assessed. All tissues were freeze dried (MicroModulyo, Edwards High Vacuum International, West Sussex, U.K.) for 24 hours and then weighted. Evans Blue dye was extracted in 2 ml formamide in a 37°C water bath for 16 hours. Absorption of extracted Evans Blue dye at 620 nm was measured with a spectrophotometer (PU 8670 VIS/NIR, Philips, Norden, Stockholm, Sweden). The concentration of Evans Blue dye was quantified by interpolation on a standard curve and expressed as ng dye/mg dry tissue. The Evans Blue dye measurement has previously been shown to highly correlate with the exudation of radio labeled albumin in guinea pig airways [25].

#### Effects of LT1 receptor and COX on early phase airway response

Three groups of guinea pigs (8-11 in each group) were sensitized with TMA. Ten days after sensitization, we evaluated the roles of LT1 receptor and COX on the early phase airway response and plasma exudation to TMA-GPSA challenge by applying ICI 198,615 (a LT1 receptor antagonist) and indomethacin (a non-specific COX-inhibitor). In this experiment, animals of group 1 were pretreated with the vehicle for ICI 198,615 and the vehicle for indomethacin 10 minutes before TMA-GPSA challenge. Group 2 received ICI 198,615 (10^-6 ^mol/kg, i.v.) and the vehicle for indomethacin, and group 3 received ICI 198,615 (10^-6 ^mol/kg, i.v.) and indomethacin (10 mg/kg, i.v.). All animals were injected with Evans blue dye, two minutes before the intratracheal instillation of TMA-GPSA. The early phase airway response and Evans blue dye exudation were evaluated [25].

### Inflammatory cells in BAL fluid

After the assessment of early phase airway response, animals were immediately sacrificed by over-dose of anaesthesia and the bronchial alveolar lavage (BAL) fluid was taken. For performing this, the thoracic cavity was opened. The systemic and pulmonary circulation were perfused through the left ventricle and the pulmonary artery with 100 ml PBS without Ca2+ and Mg2+, pH7.4, at room temperature to remove blood in the circulation. The airways were lavaged through the tracheal cannula by gentle instillation and aspiration of sterile PBS 4 ml for 5 times at room temperature. One ml BAL fluid was centrifuged at 3000 rpm at 4°C for 10 min, supernatant was collected and kept at -80°C until LTC4/D4/E4, TXB2, and PGE2 analysis. Total cell number in BAL fluid was determined in a haemocytometer using Türks solution. Cytocentrifuged preparations were stained with Giemsa and differential cell counts were carried out on 300 cells according to standard morphologic criteria.

### Measurement of LTC4/D4/E4, TXB2 and PGE2

LTC4/D4/E4, TXB2 and PGE2 in BAL fluid and airway tissue culture medium were measured with commercial enzyme immunoassay (EIA) kits (Cayman Chemical Company, MI, USA) according to the manufacturer's instructions. The concentrations of LTC4/D4/E4, TXB2 and PGE2 in BAL fluid are expressed as pg/ml BAL fluid. The productions of LTC4/D4/E4 and TXB2 in the airway tissue in vitro are dependent on the size of the airway tissue and incubation time. To standardize the measurement, the production of LTC4/D4/E4, TXB2 was therefore expressed as pg/mg protein of the airway tissue/min of incubation time. The volume of protein in the airway tissue was measured with the Bio-Rad DC Protein Assay (Bio-Rad Laboratories, CA, USA).

### Capacity of airway to produce cysLTs and TXB2

Animals of two groups (8 in each group) were sensitized with TMA. One group was exposed to PBS and one group was exposed to 0.03% TMA-GPSA on five consecutive days. Animals were sacrificed by over-dose of anaesthesia twenty-four hours after the last exposure, The thoracic cavity was opened, pulmonary and systemic circulations were perfused with PBS. Trachea, main bronchi, and intrapulmonary airways were dissected from each other and each portion was cut into 10 aliquots respectively. The airway tissue mixtures were made by randomly taking one aliquot from each portion. After equilibration by incubation in 1 ml culture medium (Waymouth MB 752/1) at 37°C for 2 hours, airway tissue was washed by removing the medium and replacing it with 1 ml fresh medium for four times. The tissue was then incubated for additional 15 min in 1 ml fresh medium complemented with either (1) 10 μl of the vehicle for calcium ionophore (DMSO, final concentration 0.2%) and 10 μl of the vehicle for arachidonic acid (AA) (95% ethanol); (2) 10 μl calcium ionophore (A23187) (final concentration 30 μM) and 10 μl of the vehicle for arachidonic acid (AA); and (3) 10 μl AA (final concentration is 10, 30, 100 μM) and 10 μl of the vehicle for A23187. The culture medium and airway tissue were collected and kept at -80°C until analysis of LTC4/D4/E4 and TXB2.

### Activity of protein tyrosine kinase Lyn after repeated allergen exposure

Animals of two groups (10 in each group) were sensitized with TMA. Group 1 was exposed to PBS and group 2 to 0.03% TMA-GPSA on five consecutive days. Twenty-four hours after the last exposure, we isolated the airway tissues and measured the activity of enzyme protein tyrosine kinase Lyn in the airway tissues with ELISA. Activity of protein tyrosine kinase lyn in the homogenate of the airway tissue was measured with a commercial ELISA kit (Pierce, Rockford, IL, USA) according to the manufacturer's instructions. The production of phosphopeptides in the tissue homogenate is dependent on the activity and amount of the protein tyrosine kinase as well as incubation time. To standardize the measurement, the activity of protein tyrosine kinase Lyn was therefore expressed as pg phosphopeptides/mg protein of tissue homogenate/min of incubation time.

### Drugs and chemicals

The following drugs and chemicals were used: ketamine hydrochloride (Park-Davis S.A., Barcelona, Spain); xylazine chloride (Bayer Sverige AB, Göteborg, Sweden); suxamethonium chloride (KabiVitum AB, Stockholm, Sweden); propranolol, pyrilamine, acetylcholine, corn oil, Waymouth MB 752/1 medium, calcium ionophore (A23187), DMSO, arachidonic acid and ovalbumin (Sigma-Aldrich Chemical Co., St Louis, USA); ICI 198,615 (Zeneca AB Sweden); indomethacin (A/S Dumex, Danmark); trimellitic anhydride (Sigma-Aldrich) and TMA-GPSA conjugate (Dept. of Occupational and Environmental Medicine, Lund University Hospital, Sweden).

### Data and statistical analysis

Data are expressed as mean ± S.E.M. for each group. Mann-Whitney *U*-test was used to test statistical significance of difference between two groups. If three or more groups were involved, Kruskal-Wallis test was used at first to ascertain that significant variance exists among the groups studied. A p-value less than 0.05 was considered significant.

## Results

### Inflammatory cells in BAL fluid

The percentage of eosinophils was significantly higher in all sensitized animals compared to non-sensitized animals. Among the sensitized animals, a single dose allergen (0.15% TMA-GPSA) exposure enhanced the percentage of eosinophils compared to PBS exposure. By contrast, the percentage of eosinophils in BAL fluid was significantly lower after repeated exposure to allergen (0.03% TMA-GPSA on five consecutive days), compared to single exposure (Table 1). The percentage of macrophages was significantly lower in all sensitized compared to non-sensitized animals, whereas the percentage of lymphocytes in sensitized and PBS exposed animals was higher than that in non-sensitized animals. There was no significant difference in neutrophil percentage between the treatment groups (Table 1).

**Table 1:** Cell composition in BAL

	Total cells (× 10^6^/lung)	Macro (%)	Eos (%)	Neutro (%)	Lympho (%)
Non-sen, PBS-expo	5.9 ± 0.9	79.1 ± 2.0	15.1 ± 1.4	4.0 ± 0.7	1.8 ± 0.3
Sen, PBS-expo	2.8 ± 0.8	57.2 ± 4.9*	31.1 ± 3.7*	7.6 ± 1.4	4.0 ± 0.6
Sen, single TMA-expo	4.3 ± 0.9	43.6 ± 3.9*	46.4 ± 3.3*#	6.9 ± 2.0	3.1 ± 0.5
Sen, repeated TMA-expo	6.3 ± 0.6	64.7 ± 3.5*	26.7 ± 2.4*§	6.0 ± 1.7	2.6 ± 0.3

The number of cells in BAL fluid in non-sensitized, PBS-exposed, sensitized PBS-exposed sensitized single TMA-exposed and sensitized repeated TMA-exposed groups. Data are expressed as mean ± SEM, Mann-Whitney *U *test, n = 11-16. *p < 0.05 non-sensitized, PBS-exposed group versus sensitized groups. # *p *< 0.05 sensitized, PBS-exposed group versus sensitized, single TMA-exposed group. §*p *< 0.05 sensitized, repeated TMA-exposed versus single TMA-exposed group.

### Cholinergic airway responsiveness

Repeated exposure of allergen (0.03% TMA-GPSA on five consecutive days) significantly enhanced cholinergic airway responsiveness to ACh compared to PBS exposure (Figure 2). There were no significant differences in baseline RL among the groups.

**Figure 2:** **Bronchial responsiveness to ACh in guinea pigs exposed to a high dose of allergen (0.15% TMA-GPSA) or repeated low dose of allergen (0.03% TMA-GPSA) on five consecutive days**. NS: non-sensitized, S: sensitized. Data are expressed as mean ± SEM, Mann-Whitney *U *test, *p = 0.03, n = 7-12 in each group.

### Early phase airway response

In non-sensitized animals, no early phase airway response was induced by intratracheal instillation of TMA-GPSA. In sensitized animals, a pronounced immediate airway response to TMA-GPSA was seen in animals previously exposed to PBS or to a single dose of allergen (0.15% TMA-GPSA). However, repeated exposure of allergen (0.03% TMA-GPSA on five consecutive days) strongly inhibited the immediate airway response to TMA-GPSA (Figure 3B).

**Figure 3:** **Time course (A) and area under the curve (AUC) (B) of the lung resistance induced by intracheal instillation of allergen (0.5%TMA-GPSA) in guinea pigs exposed to a high dose of allergen (0.15% TMA-GPSA) or repeated low dose of allergen (0.03% TMA-GPSA) on five consecutive days**. NS: non-sensitized, S: sensitized. Data are expressed as mean ± SEM, Mann-Whitney *U *test, *p < 0.01, n = 7-18 in each group.

### Specificity of early phase airway response to exposed allergen

Repeated exposure to either TMA-GPSA or OVA significantly down-regulated early phase airway response and Evans blue dye exudation to OVA in double sensitized animals (TMA and OVA) (Figure 4A, B and 4C, respectively).

**Figure 4:** **Time course (A) and area under the curve (AUC) (B) of the lung resistance and Evans blue dye (EBD) levels in airway tissue (C) induced by intratracheal instillation of OVA in double sensitized (OVA and TMA) guinea pigs**. The immediate airway response and EBD exudation to OVA challenge was inhibited by either repeated exposure to 0.03% OVA or 0.03% TMA-GPSA on five consecutive days. PIA: proximal intrapulmonary airways, DIA: distal intrapulmonary. Data are expressed as mean ± SEM, Mann-Whitney *U *test, *p < 0.05, n = 7 in each group.

### Effects of LT1 receptor and COX on early phase airway response

Combined treatment with ICI 198,615 (LT1 receptor antagonist) and indomethacin (COX inhibitor) significantly inhibited early phase airway response induced by intratracheal challenge of TMA-GPSA in sensitized animals (Figure 5A). ICI 198,615 alone or in combination with indomethacin significantly inhibited Evans blue dye exudation in all airway levels (Figure 5B).

**Figure 5:** **Immediate airflow obstruction (A) and Evans blue dye (EBD) exudation (B) after intratracheal instillation of TMA-GPSA in sensitized guinea pigs treated with vehicle, ICI 198,615 or the combination of ICI 198,615 and indomethacin**. Data are expressed as mean ± SEM, Mann-Whitney *U *test, *p < 0.05, **p < 0.01, n = 8-11 in each group.

### Levels of LTC4/D4/E4, TXB2 and PGE2 in BAL fluid and airway tissue

Repeated exposure to allergen on five consecutive days (0.03% TMA-GPSA) significantly reduced the levels of LTC4/D4/E4 and TXB2 in BAL fluid in a response to a high dose of allergen challenge (Figure 6). There was a tendency of reduction of level of PGE2 in BAL fluid after repeated allergen exposure (Figure 6).

**Figure 6:** **Production of cysLTs (LTC4/D4/E4), TXB2 and PGE2 in airway *in vivo *in sensitized guinea pigs after intratracheal instillation of allergen challenge**. Repeated exposure to allergen (0.03% TMA-GPSA on five consecutive days) prior the challenge, significantly reduced the levels of cysLTs and TXB2 in BAL fluid after intratracheal instillation of allergen. Data are expressed as mean ± SEM, Mann-Whitney *U *test, *p < 0.05, n = 8 in each group.

A high concentration of calcium ionophore (A23187, 30 μM) significantly increased LTC4/D4/E4 production in airway tissues *in vitro*, but there was no significant difference between repeated exposure to PBS and TMA-GPSA (0.70 ± 0.18 and 0.64 ± 0.12 pg/mg protein/min respectively; n = 6 in each group).

Arachidonic acid (AA) dose-dependently caused production of LTC4/D4/E4 and TXB2 in the airway tissues *in vitro*. Repeated TMA-GPSA exposure significantly enhanced the levels of LTC4/D4/E4 and TXB2 compared to corresponding PBS exposure (Figure 7).

**Figure 7:** **Production of cysLTs (LTC4/D4/E4) and TXB2 in response to arachidonic acid (AA) *in vitro***. Airway tissues from sensitized guinea pigs were stimulated *in vitro *with three different doses of AA. Arachidonic acid enhanced the production of cysLTs and TXB2 in airway tissue of animals exposed to either PBS or low dose TMA-GPSA on five consecutive days in a dose dependent manner (Spearman Rank Correlation test Rho = 0.9, p < 0.001 for cysLTs vs. doses of AA, Rho = 0.6, p < 0.03 for TXB2 vs. doses of AA). Repeated allergen exposure significantly enhanced the capacity of airway tissue to produce cysLTs and TXB2 *in vitro *compared to PBS-exposure. Data are expressed as mean ± SEM, Mann-Whitney *U *test, *p < 0.05, n = 8 in each group.

### Activity of the protein tyrosine kinase Lyn

There was no differences in activity of the protein tyrosine kinase Lyn (both cytosolic and membrane bound) in airway tissue between allergen or PBS exposure on five consecutive days (cytosolic: 1.63 ± 0.1 vs 1.57 ± 0.18; cytosolic: 1.88 ± 0.1 vs 1.63 ± 0.17 pg phosphopeptide/mg protein/min, n = 10 in each group).

## Discussion

In the present study, we have confirmed our previous findings that repeated allergen exposure increases airway cholinergic responsiveness [22]. However, we further found that repeated allergen exposure attenuates the early phase airway response to allergen and the production of LTC4/D4/E4 and TXB2 in airway during the early phase airway response.

Airway eosinophilia and bronchial hyperresponsiveness are important characteristics of allergic asthma [26]. The present study shows that sensitization alone increases the number of eosinophils in BAL fluid of guinea pigs, and that a single high dose allergen exposure (0.15%TMA-GPSA) further increases this number. Repeated exposure to allergen (0.03%TMA-GPSA on five consecutive days) does not however, significantly increase airway eosinophils compared with PBS-exposure, despite a significantly enhanced cholinergic airway responsiveness. This is in line with a previous study in Brown Norway rats showing that airway epithelial damage and bronchial hyperresponsiveness are induced after repeated exposure to low doses of allergen, without evident airway eosinophilia [22]. Thus, our experiments, together with other studies, suggest that bronchial hyperresponsiveness is not always dependent on an ongoing eosinophilic inflammation [22,27-29].

Sensitized guinea pigs, exposed to either PBS or single dose of TMA-GPSA, presented an early phase airway response to allergen. This airway response however was almost totally eliminated by repeated exposures to low doses of allergen. This reduced airway response is not due to a general reduction of contractility of the airway smooth muscle, since ACh responsiveness was higher after repeated allergen exposure (Figure 2). Furthermore, this is not either due to an increased release of endogenous bronchodilating substances since production of PGE2 also showed a tendency of decrease after repeated allergen exposure. Thus, the reduced early phase airway response, however strongly suggests a reduced mast cell responsiveness after repeated allergen exposure. Mast cell responsiveness involves the expression of the high affinity receptor for IgE (FcεRI) as well as binding of IgE receptor on the cell surface and interaction of allergen and a subsequent production and release of mediators [30]. Early phase airway response is mainly mediated by histamine, cysLTs, and probably also TXA2 released from mast cells during the response to allergen challenge. These mediators can induce both airway constriction and airway plasma exudation [3,12,14].

To further delineate if the reduced response to TMA challenge seen in the repeatedly exposed animals is due to a tolarized effect to the TMA-GPSA allergen. We sensitized guinea pigs with two allergens (TMA and OVA), and exposed animals to one of the two allergens and thus evaluated the early phase airway response and plasma exudation. Our experiment revealed that repeated exposure to each of allergens (either TMA-GPSA or OVA) inhibited early phase airway response and Evans blue dye exudation. Therefore, this allergen-unspecific inhibition of airway responses is thus not likely related to allergen-IgE interaction but rather suggests a mediator(s) mechanism.

Early phase airway response to allergen is closely related to mediators such as histamine, cysLTs, and TXA2. However, our data reveal a histamine independency, since in the present study pretreatment with a H1 receptor antagonist showed no differences between groups. Thus, to further elucidate the role of cysLTs and TXB2 in our guinea pig model, we measured the levels of these mediators in BAL fluid after allergen challenge. Our data show that after repeated exposure to allergen, the levels of cysLTs and TXB2 in the airways are significantly reduced. Thus, this could at least in part be the explanation for the reduction of early phase airway response after repeated allergen exposure.

In asthmatic patients, the concentrations of cysLTs and TXA2 are increased in plasma, urine and BAL fluid during asthma exacerbation and after experimental allergen challenges [8-11,31]. To investigate whether cysLTs and TXB2 work in same way in our guinea pig model as in humans, we applied ICI 198,615 (a LT1 receptor antagonist) and indomethacin (a non-specific COX inhibitor) to sensitized guinea pigs before allergen challenge. A combined treatment of ICI 198,615 and indomethacin attenuated early phase airway response and plasma exudation in response to TMA-GPSA challenge. This suggests an important role of arachidonic acid metabolites in early phase airway response to allergen challenge in guinea pigs, resembling the acute allergic bronchoconstriction in humans [12,14].

To further understand whether the reduction of cysLTs and TXB2 to repeated allergen challenge is due to a decrease of the activity of 5-LO and COX2 pathways, we measured the levels of these mediators in isolated airway tissues from sensitized and repeatedly TMA-exposed guinea pigs, in response to exogenously applied arachidonic acid. The production of LTC4/D4/E4 and TXB2 in vitro was significantly enhanced in the airways of repeatedly TMA-exposed guinea pigs, consequently, suggesting an up-regulation of 5-LO and COX pathways. Furthermore, we found no reduction of LTC4/D4/E4 production in airway tissues incubated with a high dose of calcium ionophore. These data suggest that there is no reduction of substrate for 5-LO after repeated allergen exposure. Taken together, these data argue against a reduction in arachidonic acid mediator production via down-regulation of the enzymes.

To further investigate the mechanism behind the reduced production of cysLTs and TXB2 in airway after repeated allergen exposure, we measured the activity of protein tyrosine kinase Lyn, which is an intracellular signaling molecule downstream FcεRI, and may regulate production of cysLTs and TXB2. Allergen-induced aggregation of FcεRI on mast cell activates tyrosine kinase Lyn that binds to the FcεRIβ-chain under resting conditions [32]. Once activated, Lyn phosphorylates the tyrosine residues in the FcεRIγ-chain and recruits other signal molecules and finally activates 5-LO and COX [16,17]. However, in the present study we could not find any deduction of Lyn activity after repeated allergen exposure compared to PBS exposure, thus implicating the involvement of other intracellular signaling molecules in regulating this response. One hypothesis that remains to be investigated is that repeated allergen exposure may down-regulate the expression of IgE-receptor and thus reduce mast cell responsiveness in general, but solid techniques to quantify guinea pig IgE-receptor are missing. Another hypothesis might be an altered balance between the IgE-receptor (FcεRI) and inhibitory receptors on mast cells, such as FcγRII in response to repeated low dose allergen exposure. Thus, studies in rodent mast cells suggest that coligation of FcγRII with FcεRI results in a downregulation of IgE-FcεRI mediated inflammatory mediator release [33].

Our current findings may have clinical implications. Patients presenting recurrent and reversible airflow obstruction but shows low or no response to allergen challenge in laboratories may actually have an allergen driven airway disease. Patients' airway response to allergen may have been down-regulated by repeated allergen exposure, such as house-dust mite, animal dander or some occupational allergen [34]. Thus, in a previous clinical study, we have showed that repeated low dose allergen exposure attenuates the late phase airway response to allergen, despite existing bronchial hyperresponsiveness [23]. This suggests that reduced allergic response to allergen by repeated allergen exposure is present not only in animal, but also in humans.

In summary, the current study indicates that in sensitized guinea pigs, repeated exposure to allergen inhibits allergen induced early phase airway response despite existing non-specific bronchial hyperresponsiveness, possible via reduced cysLTs and TXB2 production. These findings might result from mast cells being less responsive after repeated allergen exposure. Thus, reduced production of cysLTs and TXB2 may reflect an impaired intracellular mast cell signaling and could explain the mechanisms of the reduced allergen induced early phase airway response.

## Abbreviations

EAR: Early asthmatic responses; AUC: Area under the curve.

## Competing interests

The authors declare that they have no competing interests.

## Authors' contributions

JL conceived and coordinated the study. ZHC and MS performed experiment, analysis and interpretation of data. ZHC and MR wrote the manuscript with significant input from JL and MS. All authors read and approved the final manuscript.
